The article "PPARs and Adipose Cell Plasticity" was published in 2007. Journal: PPAR Res.

# PPARs and Adipose Cell Plasticity

**DOI:** 10.1155/2007/68202

**Published:** 2007-07-10

**Authors:** Louis Casteilla, Béatrice Cousin, Mamen Carmona

**Affiliations:** ^1^IFR 31, Institut Louis Bugnard, CNRS/UPS UMR 5241, 31432 Toulouse Cedex 4, France; ^2^Laboratorio de Diabetes y Obesidad Experimentales, Institut d'Investigacions Biomèdiques August Pi i Sunyer (IDIBAPS), Hospital Clínic de Barcelona, Villarroel, 170, 08036 Barcelona, Spain

## Abstract

Due to the importance of fat tissues in both energy balance and in the associated disorders arising when such balance is not maintained, adipocyte differentiation has been extensively investigated in order to control and inhibit the enlargement of white adipose tissue. The ability of a cell to undergo adipocyte differentiation is one particular feature of all mesenchymal cells. Up until now, the peroxysome proliferator-activated receptor (PPAR) subtypes appear to be the keys and essential players capable of inducing and controlling adipocyte differentiation. In addition, it is now accepted that adipose cells present a broad plasticity that allows them to differentiate towards various mesodermal phenotypes. The role of PPARs in such plasticity is reviewed here, although no definite conclusion can yet be drawn. Many questions thus remain open concerning the definition of preadipocytes and the relative importance of PPARs in comparison to other master factors involved in the other mesodermal phenotypes.

## 1. INTRODUCTION

Adipose tissues have long been associated with the invasive prevalence of obesity and metabolic disorders. Recent advances have focused the attention on the presence of intriguing cells able to differentiate towards various phenotypes and recall the old use of fat in plastic and reconstructive surgery [1–3]. Two rather distinct medical and scientific domains share these perspectives but irrespective of field, a good understanding of adipogenesis is absolutely requisite to manipulating and controlling adipocyte differentiation. This point is emphasized by the fact that adipocyte differentiation belongs to the mesenchymal stroma or stem cell hallmark. We thus should consider that any of these cells can acquire the adipocyte phenotype depending on its environment. In this view, peroxysome proliferator-activated receptor (PPAR) family of transcription factors appears to be a key and unavoidable actor.

After a brief overview on adipose tissues, this review will focus on the importance of PPARs and PPAR*γ* in particular in adipose-derived cell phenotype and plasticity.

## 2. ADIPOSE TISSUES:WHAT ROLE DO PPARS PLAY?

### 2.1. Adipose tissue or adipose tissues?

Three functionally different types of adipose tissues are described in mammals: brown adipose tissue (BAT), white adipose tissue (WAT), and bone-marrow adipose tissue (BMAT) [4–6].

BAT and WAT participate differently in energy balance and homeostasis. BAT is heavily involved in nonshivering thermogenesis (cold and diet-induced thermogenesis). In contrast, WAT is mainly involved in energy storage and is now considered an endocrine organ [4–7]. Brown and white adipocytes similarly display lipogenesis, triglyceride accumulation, and lipolysis, but brown adipocytes are also specialized in energy dissipation in the form of heat. These cells are smaller than white adipocytes, contain abundant mitochondria and highly express the uncoupling protein-1 (UCP-1) [8]. This protein, by uncoupling ATP synthesis from the respiratory-chain function, subsequently promotes the dissipation of energy as heat [9]. It is noteworthy that only 40%–60% of the whole cell population in BAT as well as in WAT is composed of mature adipocytes. Endothelial, haematopoietic cells, and adipocyte precursors, the so-called preadipocytes, or adipose-derived stromal cells (ASCs) are also found in adipose tissues [10]. It has long been known that adipocyte precursors are present throughout adulthood and can proliferate and/or be recruited depending on physiological or physiopathological situations [7]. BAT and WAT develop at specific and different locations and WATs various locations also determine its different metabolic and molecular features [11, 12].

In contrast to brown and white adipocytes, the role of medullar adipocytes has been poorly investigated and is not well-understood [5]. The number and size of adipocytes seem to be inversely correlated to haematopoietic activity in bone marrow based on the physiological or physiopathological situation. Nevertheless, it is noteworthy that many scattered adipocytes are observed in active haematopoietic bone marrow. Highly similar gene expression has been described between human subcutaneous and medullary mature adipocytes, suggesting that medullary adipocytes may share some of the functions exhibited by subcutaneous and visceral adipocytes [13].

Beside the physiological anatomy of adipose tissues, ectopic location of adipocytes is also observed in degenerative tissues. The origin of these adipocytes infiltrating the degenerative tissues is still unclear.

### 2.2. PPARs and white adipocyte differentiation

As usual in any differentiation program, a subtle balance and interconnection exist between cell cycle and commitment to adipocyte differentiation. In this context, overexpression of both C/EBP*α* and PPAR*γ*, mediates the cell cycle arrest after clonal expansion. Indeed, PPAR*γ* induces cell cycle withdrawal by the inhibition of the transcription factor E2F/DP DNA-binding activity via downregulation of the protein phosphatase 2A (PP2A) [14]. In the opposite, E2Fs trigger clonal expansion, and terminal adipocyte differentiation through regulation of PPAR*γ* expression [15]. In the same manner, p107 protein belonging to retinoblastoma family is also involved in regulating PPAR*γ* and its recovery into deficient cells reduces adipocyte differentiation through the downregulation of PPAR*γ* activity [16]. The potency of PPAR*γ* and its interplay with cell cycle is illustrated by a report studying liposarcoma cells. Treating cells from these aggressive tumours with ligands for both PPAR*γ* and the retinoid X receptor (RXR) forces their terminal differentiation [17]. Indeed, the antiproliferative activity of PPAR*γ* is now investigated to limit and treat tumour cell proliferation although several PPAR*γ* ligand-mediated antiproliferative effects act through a complexity of PPAR*γ*-independent mechanisms [18]. Nevertheless, this antigrowth effect seems to be specific to cell type because PPAR*γ* activation promotes the proliferation of neural stem cells [19], instead of their differentiation.

The crucial role for PPAR*γ* as a dominant regulator of white-adipocyte differentiation is now well documented and largely reviewed [20, 21]. It interplays with several other nuclear factors such as CAAT Enhancer Binding Protein (C/EBP) and Sterol regulatory element-binding proteins (SREBP) families and numerous coactivators or corepressors. The use of genetic ablated cells demonstrates that while the lack of C/EBP*α* can be overcome by the overexpression of PPAR*γ*, the opposite does not hold true that PPAR*γ* is absolutely required for the adipogenic program [22]. During this program, the expression of both factors is interdependent not only in promoting adipocyte differentiation but also in sustaining and maintaining the fully differentiated adipocyte phenotype. Any signal able to modulate one or the other of both transcription factors subsequently induces change in adipocyte differentiation. Thus, insulin/IGF-I signalling modulates adipogenesis by the upregulation of PPAR*γ* expression via the insulin/IGF-I receptor-AktSH2-B-Foxo1- pathway [23].

Whereas PPAR*γ* was described as a factor involved in white adipocyte differentiation, PPAR*α* and *δ* were described for their role in fatty acid oxidation in several tissues including adipose tissue [24–27]. However, gain-of-function experiments suggest that both PPAR*δ* and PPAR*γ* isoforms are required to facilitate maximal lipid accumulation and differentiation during white adipogenesis [28].

As PPAR*γ* stimulates white adipogenesis, its negative control inhibits this process. In this way, hypoxia-mediated inhibition of adipogenesis can be partly explained via the repression of PPAR*γ* expression by the hypoxia-inducible factor-1 (HIF-1)-regulated gene DEC1/Stra13, a member of the Drosophila hairy/enhancer of split transcription repressor family. Similarly, the inhibition of adipogenesis by cytokines is mediated via the repression of PPAR*γ* function through kinase cascade [29, 30]. It has also been demonstrated that the constitutive expression of GATA-2 and GATA-3 resulted in a decrease in PPAR*γ* expression and a consequent inhibition of adipocyte differentiation [31].

### 2.3. Preadipocytes, circulating cells, and PPARs

The first report in this field was published in 2005. Its authors described a circulating human cell population able to differentiate towards adipocytes when cultured under adipogenic conditions. Moreover, these human progenitors engrafted and formed adipose tissue following injection into SCID mice [32]. This report is now supported by a recent investigation suggesting that new fat cells arise not only from resident precursor cells within the tissue, but also from other sources, such as BM-derived circulating progenitor cells. One difference between both reports is the nature of the newly-formed adipocytes. In the first study, unilocular white adipocytes were observed whereas in the second, mutlilocular cells, expressing low levels of UCP1, were detected. In this work, the appearance of bone-marrow-derived adipocytes in the fat pad is triggered by PPAR*γ* ligand [33]. No explanation is proposed for this effect of PPAR*γ* ligand, although it appears to be at least partly a specific mechanism because this phenomenon is not totally reproduced by a high fat diet. Obviously, the underlined mechanisms and the relevance of such observations need further investigation, but could participate in the ectopic emergence of fat cells through the local recruitment of circulating adipocyte progenitor cells.

### 2.4. Role of PPARs in white and brown adipocytes

The relationship between brown and white fat is complex because besides the typical interscapular brown adipose tissue, an extensive analysis of the different fat deposits revealed that scattered brown adipocytes are present in any white adipose depot also in primates [34, 35]. Furthermore, brown fat can extensively change into white-like fat and conversely, according to physiological or physiopathological situations and the species [36]. These properties led us to use the term “plasticity of adipose tissue.” The main pitfall is that a lack of uncoupling protein-1 (UCP-1) expression is taken as the gold standard for white fat and no positive marker is yet characterized to clearly identify white adipose phenotype. Thus, with the present knowledge, it is not possible to determine whether brown adipocytes can be transformed into white-like adipocytes with different metabolic properties (termed masked brown adipocyte) or into true white fat cells. The establishment of different preadipocyte cell lines and the use of primary culture favor the existence of distinct precursor cells [4]. First depending upon the origin of cultured cells (i.e., from brown or white fat) a corresponding brown or white mature phenotype is obtained [37]. Second, genetic manipulations allowing irreversible labelling of brown adipocytes show that they do not convert into white adipocytes during normal mouse development [38]. Third, no differentiation of pluripotent mouse embryonic stem cells into brown adipocytes even after PPAR*γ* activation take place whereas white phenotype can be easily obtained [39]. In this regard, it is noteworthy that brown adipocyte is the only cell type that coexpresses high levels of the three PPAR subtypes. Furthermore, PPAR*α* and PPAR*γ* are strictly subjected to opposite regulation by retinoids in brown fat, supporting the notion of specific physiological roles of each transcription factor in controlling brown fat differentiation and thermogenic activity [40]. A further step was undertaken when PGC-1, for PPAR*γ* coactivator 1, was identified in brown fat. Initially claimed as a specific factor to brown fat, it was proposed to be a coactivator involved in brown versus white adipocyte differentiation. This coactivator has been shown to control a subset of genes involved in mitochondrial activity and biogenesis [21, 41]. This is consistent with the adenovirus-mediated expression of human PGC-1*α* that increases the expression of UCP1, respiratory chain proteins, and fatty acid oxidation enzymes in human adipocytes differentiated in primary culture [42]. Nevertheless it appears that this protein displays numerous functions in many tissues, all of them related to mitochondrial function [43]. Other factors have been proposed to be central switches for white to brown adipocyte differentiation, including the retinoblastoma protein [44] and the corepressor RIP140 [45].

## 3. PPARS AND MESODERMAL FATES

Although, it is well admitted that adipose cells arise from mesodermal origin, the exact origin of adipocyte precursors is not well defined as illustrated by the recent work on circulating adipose precursors [32]. Recently, it appears that cells named previously preadipocytes can differentiate towards various mesodermal origins [46–48]. These cells were thus named adipose derived stromal cells (ADSC). Conversely, it seems that adipocyte phenotype could be obtained from different cells including myoblasts [49]. PPARs may thus be involved in the preferential cell commitment towards one or the other lineage and/or in maintaining pluripotency. These aspects are discussed in the second part of this review.

### 3.1. Adipocyte versus osteogenic potential

Many reports have demonstrated that adipocytes and osteoblasts share a common precursor. Osteoblastic genes are expressed in cell lines able to differentiate towards adipocyte. Bipotent cells with features specific to both osteoblasts and preadipose cells have been cloned from bone marrow [50] and more recently from human adipose tissue [47, 48, 51, 52]. Recently, Birk et al. have shown that the 3T3-F442A preadipocyte clonal cell line differentiate into osteoblasts [53]. It has also been reported that stromal colonies, either undifferentiated or differentiated into mature adipocytes, are able to give rise to osteogenic cells when transplanted in intraperitoneal diffusion chambers. These observations suggest that stromal cells, first differentiated along the adipogenic lineage, are able to dedifferentiate and then to redifferentiate in an osteoblastic phenotype.

Several transcription factors, such as PPAR*γ* and Runx2, have been proposed as playing a critical role in the commitment of bipotent stem cells towards the adipogenic or the osteogenic lineages [54]. However, it has to be noted that the effect of genes of interest are often investigated in different cell lines already committed in either one or the other lineage, making dubious their role in the regulation of the commitment of a multipotent stem cell. For example, ectopic overexpression of adipogenic transcription factors such as PPAR*γ* induces transdifferentiation of mouse osteoblastic MC3T3-E1 cells into mature adipocytes [55]. A unique investigation really addressed the issue of the commitment of stem cells on embryonic stem (ES) cells. In this report, the authors transiently suppressed PPAR*γ* expression. This genetic manipulation directs ES cells into an osteoblastic lineage suggesting that PPAR*γ* can be considered a proadipogenic as well as an anti-osteoblastic factor [56]. The role of the transcription factor deltaFosB has been investigated in further detail. Overexpression of deltaFosB under the control of a promoter-driving transgene both in osteoblasts and adipocytes led to increased bone mass and decreased adipocyte formation. Given the assumption of a reciprocal development of both lineages, it has been proposed that differentiation into one cell type could be a consequence of the action of deltaFosB in the other [57]. More recently, elegant experiments from the same group generating transgenic mice that express deltaFosB in a bone-specific manner, led the authors to conclude that the change in osteoblast and adipocyte differentiation results from independent cell-autonomous mechanisms [58]. Therefore, factors playing a role in the switch of stem-cell differentiation towards the adipogenic or osteogenic lineages remain to be definitively identified. The 14-3-3-binding protein, TAZ (transcriptional coactivator with PDZ-binding motif), which coactivates Runx2-dependent gene transcription while repressing PPAR*γ*-dependent gene transcription could be also involved [59].

### 3.2. Myoblast and Preadipocyte

The deciphering and understanding of myogenesis is far beyond our current understanding of adipogenesis, but both programs are closely linked by their mesodermal origin and the well-described emergence of adipocytes in denervated muscle. From such observations, the question of a putative role of PPARs in directing cell fate towards one of the differentiation programs seems reasonable. As described for fibroblasts, overexpression of PPAR*γ* or activation through its ligands in satellite cells transdifferentiates myoblasts towards the adipogenic phenotype. This characteristic is shared by the other key adipogenic factor, C/EBP*α* [60]. This transdifferentiation was observed for myoblasts in all mammals and during the whole development [49]. In addition, the activation of PPAR*δ* abolishes the development of multinucleated myotubes while inducing the expression of PPAR*γ* gene. Loss and gain function experiments are consistent with a role for PPAR*δ* as an inducer of transdifferentiation into adipocyte-like cells, which precedes and triggers PPAR*γ* expression [61].

On the other hand, PPAR*γ* can be controlled by Wnt proteins and especially Wnt 1 and Wnt-10b that govern adipogenesis. Indeed, PPAR*γ* as well as C/EBP proteins is inhibited by Wnt signalling, which in turn maintains preadipocytes in an undifferentiated state. When Wnt signalling in preadipocytes is prevented by the overexpression of Axin or dominant-negative T-Cell Factor-4 (TCF4), these cells differentiate into adipocytes. These results are strengthened by the fact that the lack of Wnt signalling also induces transdifferentiation of myoblasts into adipocytes [62]. However, the relationship between Wnt signalling and PPAR*γ* seems to be complex because the impairment or activation of Glycogen Synthase Kinase-3*β* (GSK3*β*)/*β*-catenin only affects a subset of PPAR*γ*-dependent genes [63].

Finally, it has been suggested that myostatin, a potent negative regulator of skeletal muscle growth member of the transforming growth factor beta (TGF-*β*) family, blocks adipocyte differentiation via down regulation of PPAR*γ* in 3T3-L1 [64]. However, recent data reports that in pluripotent C3H10T1/2 cell line, myostatin treatment may promote the differentiation of multipotent mesenchymal cells into the adipogenic lineage and inhibit myogenesis [65, 66].

### 3.3. Preadipocytes and macrophages

Analysis of the literature lined out that adipocyte and monocyte/macrophage lineages have many features in common including aP2 and PPAR expression. More surprisingly, we demonstrated that preadipocytes efficiently phagocytoze yeasts and apoptotic bodies in a similar manner, albeit to a lesser extent, than specialized phagocytic cells such as macrophages [67, 68]. This suggests the involvement of adipocyte progenitors in tissue remodelling and plasticity through the discarding of apoptotic bodies. A profiling analysis between adipocyte and macrophage lineages expanded the known similarities between these cell phenotypes [69]. Finally, preadipocytes can be very rapidly converted into macrophage-like cells when injected into the peritoneal cavity, considered a likely environment for supporting macrophage phenotype [69]. The rapidkinetics of change suggests a transdifferentiation process and/or a stronger lineage relationship between adipocyte progenitors and macrophages than expected. Since only 80% of the macrophages come from bone marrow in obesity [70], one could thus postulate that the remaining 20% of adipose-tissue-resident macrophages derive from preadipocytes. According to the importance of PPAR*γ* to direct cells towards adipocyte differentiation, it is reasonable to wonder if PPARs could be involved in such plasticity.

PPAR*γ* is expressed at low levels in circulating monocytes and its expression increases significantly upon differentiation to macrophages, including in the foam cells of atherosclerotic lesions. Numerous studies have thus focused on its role in macrophage metabolism and activation and its possible involvement in the process of atherosclerosis. These studies have provided evidence supporting a role of PPAR*γ* in both lipid uptake and lipid efflux pathways in macrophages [71]. The fact that PPAR*γ* could influence both lipid uptake and efflux raised the question of whether the net effect of PPAR*γ* ligands on macrophages within an atherosclerotic lesion would be to promote or impede foam cell formation. PPAR*γ* is not essential for myeloid development or for mature macrophage functions, such as phagocytosis and inflammatory cytokine production [72]. It is also a negative regulator of macrophage activation and inhibits macrophage production of inflammatory cytokines, although some of this activity may not be mediated by PPAR*γ* [73]. In addition, PPAR*γ* agonists inhibit foam-cell formation in vivo [74]. However, such an effect could be cell-type dependent [75]. Although PPAR*γ* seems fundamental in preadipocyte and macrophage biology, adipocytes and foam cells are probably distinct cell types and thus far no study has described a potential role of PPAR*γ* in the differentiation of preadipocytes into macrophage-like cells.

## 4. CONCLUSION

The importance and the role of PPARs in adipogenic process is definitively demonstrated and brought numerous new insights in our understanding of adipogenesis but many questions remain open concerning the definition of preadipocytes and the relative importance of PPARs compared to other master genes involved in other mesodermal phenotypes. Altogether, the negative regulation of several master proteins involved in other mesodermal differentiation programs suggests that at least PPAR*γ* can play its role only when all negative regulators are missing. This could suggest that preadipocyte status results from a default pathway.

Similarly, the tissue origin of preadipocytes is now challenged and needs to be clarified because it can help to build a more dynamic view of adipose tissue development and the role of PPAR proteins.
